# Efficacy and Safety of Moxibustion for Menopausal Obesity: A Multicentre, Randomized, Controlled Trial Protocol

**DOI:** 10.1155/2022/9255017

**Published:** 2022-08-04

**Authors:** Benlu Yu, Wei Huang, Yingrong Zhang, Jiajie Wang, Chen Xia, YanJi Zhang, Hongjie Xia, Yaxin Hu, Yingyue Rao, Zhongyu Zhou

**Affiliations:** ^1^College of Acupuncture and Orthopedics, Hubei University of Traditional Chinese Medicine, No. 01 Tanhualin, Wuchang District, Wuhan 430060, Hubei, China; ^2^Department of Acupuncture, Hubei Provincial Hospital of Traditional Chinese Medicine affiliated to Hubei University of Traditional Chinese Medicine, No. 4 Garden Hill, Liangdao Street, Wuchang District, Wuhan 430061, Hubei, China

## Abstract

*Background*. In the past, moxibustion has been widely used to treat endocrine system disorders, but evidence of its effectiveness is scarce at this point. The aim of this multicenter, randomized, controlled trial is to evaluate the efficacy and safety of treating menopausal obesity with moxibustion. *Methods/Design*. There are six centers taking part in this randomized, controlled, parallel trial. A total of 216 patients with menopausal obesity will be randomly divided into two equal groups: the “moxibustion for harmonization of Yin and Yang” group and the gentle moxibustion group. A 12-week study period with moxibustion will be preceded by a 1-week baseline, followed by a 12-week follow-up. We will conduct an interim analysis to determine whether or not the treatment is efficacious and safe after 216 participants have completed a 12-week treatment period. Evaluations will be conducted at weeks 0, 4, 8, 12, 18, and 24. The main outcome is waist circumference (WC), and the rate of WC reduction will be compared to the baseline. An intention-to-treat analysis will be performed with a two-sided *P* value of <0.05 considered significant. Participants who withdraw from the trial will be analyzed according to the intention-to-treat formula (ITT). *Discussion*. These results will be used to support selecting the right moxibustion prescription and guiding the improvement of clinical efficacy. This trial will provide convincing evidence of moxibustion's effectiveness and safety in the treatment of obesity by “moxibustion for harmonization of Yin and Yang,” which will be conducive to the promotion and clinical application of the theory of “moxibustion for harmonization of Yin and Yang.” *Trial Registration*. This trial is registered with Clinical Trials.gov: NCT04943705 (registered on June 27, 2021).

## 1. Introduction

Obesity is a multifactorial condition caused by genetic, physiologic, behavioral, sociocultural, and environmental factors that lead to an imbalance between energy consumption and expenditure over a long period of time [1]. According to the Global Burden of Disease Obesity Collaborators, 603.7 million adults worldwide suffer from obesity [2], and the global prevalence of overweight or obesity ranges from 39% to 49% [3], with morbidity doubling between 1980 and 2015 in 73 countries. In addition to significantly decreasing the quality of life of patients, obesity is associated with an increased risk of illness (such as diabetes, hypertension, and cardiovascular disease) and mortality [1, 4, 5]. Moreover, it causes mental illnesses (e.g., depression, unwarranted stigma, and schizophrenia) and increases health care costs in countries all over the world [6–8]. Menopause is characterized by an increase in FSH levels [9]. This is a time when women are susceptible to gaining a great deal of visceral fat due to increased glucocorticoid secretion and increased glucocorticoid secretion, among other factors [10, 11]. A woman who is obese at menopause may also have an increased risk of developing breast cancer, endometrial and colon cancer, type 2 diabetes, and cardiovascular disease [12]. In a meta-analysis [13], obesity is associated with a 25% to 30% relative increase in breast cancer-specific and overall mortality among menopausal women.

At present, the main intervention methods for obesity include lifestyle intervention, western medicine treatment, bariatric surgery, and traditional Chinese medicine therapy [14]. A simple diet and exercise method is often difficult to adhere to and easy to rebound [15]. Western drugs for weight loss need clear indications, and long-term safety studies for weight loss drug therapy are lacking [16]. Multiple randomized controlled trials have reported bariatric surgery's effectiveness in treating obesity, but it also carries a greater risk of cardiovascular disease and mortality and is costly [17]. Consequently, seeking safe and effective therapies for menopause obesity prevention and control has become an increasingly important concern.

Moxibustion, as a green therapy for weight loss because of its safe operation, outstanding curative effect, low cost, and good patient compliance, has become a popular treatment option for obese patients in recent years. Numerous studies indicate that moxibustion is efficient in relieving menopausal symptoms by enhancing the immune system and altering the amounts of neurotransmitters in the central nervous system through repeatedly stimulating acupoints[18, 19]. As far as we know, by applying moxa to warm acupoints and body areas, moxibustion can promote a smoother flow of qi and blood in the human body[20]. This increases blood circulation generally, which has the benefits of illness prevention and health care. By activating beige fat via the HSF1-A2B1 transcriptional axis, moxibustion can be utilized to treat obesity through local thermal stimulation[21]. It is acknowledged that menopausal obesity is caused by the imbalance of Yin and Yang according to the theory of etiology and pathogenesis of traditional Chinese medicine. Based on this, our research group innovatively apply “moxibustion for harmonization of Yin and Yang” to treat menopause obesity, so as to restore the balance between Yin and Yang. Compared with ordinary moxibustion, “moxibustion for harmonization of Yin and Yang” achieves coverage from point to surface. As for moxibustion quantity, it has a wider range of treatment and higher comfort. The frequency of moxibustion is usually once a week, which saves the time cost of patients' medical treatment and is more convenient. In sequence and position of moxibustion, double-sided moxibustion with the Yang side before the Yin side promotes spontaneous harmonization of Yin and Yang. However, for menopausal obesity, due to hormone levels, psychological state, and other reasons, the curative effect of moxibustion is often unable to be unified. There have not been many studies comparing various moxibustion techniques side by side to see how effectively they vary.

The Study of Women's Health Across the Nations (SWAN) [22], an observational cohort of menopausal female followed for over a decade, have suggested that after the onset of menopause, due to estrogen loss, women often continue to have bone loss, disrupted energy balance, and reduced physical activity and further accrue visceral fat, resulting in obesity [23]. Modern studies have shown that [24, 25] moxibustion can improve immunoglobulin and reduce proinflammatory cytokines and promote energy metabolism. It also has the effect of regulating nerves, anti-inflammatory properties, enhanced immunity, and accelerated metabolism.

Therefore, this multicenter randomized controlled research is on the variations in effectiveness between the two moxibustion prescriptions for treating menopausal obesity by assessing the safety, efficacy, and health economic evaluation of the “moxibustion for harmonization of Yin and Yang” compared to the gentle moxibustion, in order to increase the therapeutic impact and give high-quality evidence-based evidence for a better choice of moxibustion prescription.

## 2. Methods and Design

### 2.1. Objectives

This study aims to (1) assess the effectiveness and security of moxibustion in the treatment of menopausal obesity; (2) compare the safety, efficacy, and health economic evaluation of different moxibustion methods for treating menopausal obesity, so as to optimize the prescription of moxibustion; and (3) investigate the effect of moxibustion in ameliorating the metabolism and relieving symptoms of menopause.

### 2.2. Study Design

This will be a multicenter, randomized, controlled, two-arm clinical trial, where 216 participants will be randomized at a ratio of 1 : 1 to two groups (108 participants per group). There are six academic hospitals in China where this study will be carried out: Hubei Provincial Hospital of TCM, Shanxi Provincial Hospital of TCM, Shenzhen Baoan Hospital of TCM (Group), Xiamen Hospital of TCM, Jiangsu Provincial Hospital of TCM, and the First Affiliated Hospital of the Hunan University of TCM. A 12-week treatment phase plus a 12-week follow-up period make up the 24-week duration of this research. If they are qualified for the study, each participant is required to keep a diet and exercise diary for the whole research cycle. All participants will receive 12 weeks of individual treatments in two groups: the “moxibustion for harmonization of Yin and Yang” will be administered once every 1 week, 60 minutes each time; the gentle moxibustion will be administered 3 times a week, 20 minutes each time. Outcomes will be assessed at the beginning, at the conclusion, and during the follow-up period. The Standard Protocol Items: Recommendations for Intervention Trials (SPIRIT) [26] are utilized in the protocol, which is based on the Standards for Reporting Interventions in Clinical Trials of Acupuncture (STRICTA) [27](Additional file 1).  Figure 1 provides a summary of the trial's design.

### 2.3. Recruitment

we will create a public recruiting advertisement in newspapers, posters, WeChat, or the Internet and seek any patients who fit the requirements. Patients' eligibility to take part in this study will be decided by the doctor. Each patient will have enough time to decide whether or not to take part in the research. And each participant will be required to sign a freely completed written informed consent form. It informs patients about connected clinical research in terms that patients or their legal representatives may comprehend, including explanations of the study purpose, research technique, and procedure.

### 2.4. Participants

#### 2.4.1. Inclusion Criteria

(1) Obesity diagnostic criteria: waist circumference ≥ 80 cm and BMI ≥ 25 are the criteria listed in the Comprehensive Medical Management Guidelines for Obese People jointly published by the American Society of Clinical Endocrinologists (AACE) and the American College of Endocrinology (ACE) in May 2016 [28]
(2) Menopausal syndrome diagnostic criteria: refer to “Obstetrics and Gynecology” [29]and the China Association for Traditional Chinese Medicine's recommendations for the diagnosis and treatment of menopausal syndrome in 2020 [30]:
  ① women's age is 40–60
  ② The menstruation is out of the regularity, and the menstrual cycle appears >7 days, but <2 months, or the menopause time >2 months, rule out the menopause caused by other reasons
  ③ There are manifestations of menopausal syndrome with kidney Yin and Yang deficiency: before and after menopause, menstrual disorders, dark or light red menstruation, sometimes hot, sometimes chills; spontaneous sweating, night sweats, dizziness, tinnitus, insomnia, forgetfulness, cold back pain, heel pain, swelling, loose stools, frequent urination; pale tongue, white fur, heavy, and weak pulse
  ④ Serum FSH>10IU/L
(3) Having not used any hormone-related or weight-loss-related medications in the previous 3 months
(4) Being the ability to fully comprehend and willingly sign informed consent

#### 2.4.2. Exclusion Criteria

1. Unexplained vaginal bleeding, or unnatural menopause
2. History of using hormone replacement treatment or other medications for the condition within the previous 3 months
3. Respiratory illnesses, heart, liver, and renal problems, as well as severe organic and endocrine diseases
4. Hypothalamic lesions, hypothyroidism, glucocorticoid medication, and other conditions can produce secondary obesity
5. Organic illnesses of the uterus, such as polycystic ovary syndrome, malignant tumors, severe cervical erosion following complete hysterectomy, and so forth
6. Contraindications to moxibustion include moxibustion intolerance, skin allergies, scarring, and other significant skin illnesses
7. Inability to adhere to therapy due to poor compliance

#### 2.4.3. Withdrawal from the Study

1. Pregnancy or other diseases are found during treatment, or serious adverse reactions and complications occur, and a specialist physician at each center decides to terminate the patient's participation in the trial
2. Combines the treatment methods prohibited by this study or changes the specified treatment method halfway
3. Poor compliance and unable to implement treatment in accordance with the prescribed test protocol
4. Participant's decision to withdraw from the study

### 2.5. Randomization and Allocation Concealment

To complete the randomization, we will utilize an online or messaging system run by a clinical information management system (Beijing Shuanghua Science and Technology Development Co, Ltd. China). When a subparticipant-recruiting center's staff accepts an eligible menopausal obesity patient, the patient's name, gender, age, and medical history are entered into the central randomization system. The acupuncturists will then be allocated a random number and an identity code that are unique to each participant. The allocation number will be kept secret from all participants.

### 2.6. Blinding

Throughout the study, participants will be kept in the dark about their group assignment. They will listen to an explanation that they will undergo “moxibustion for harmonization of Yin and Yang” or “gentle moxibustion.” The assessor, data recorder, acupuncturist, and statistician will all work independently; the randomization staff and acupuncturist will be aware of the allocation information, but the assessor and statistician will stay blind to it throughout the trial. To avoid the interchange of study information, each participant will be treated independently. In the event of withdrawal, the study research assistant would present the participant with the pertinent information, which would include the individual's treatment assignment and outcome data.

### 2.7. Interventions

#### 2.7.1. Lifestyle Modification

Both groups of patients get lifestyle intervention, with the following suggested living habits [31]: all individuals weighing 113.6 kg (250 lb.) will be provided a diet of 1200 to 1499 kcal/day consisting of standard foods with roughly 20% to 35% kcal from fat, 15% to 20% kcal from protein, and the remaining from carbohydrate. Those weighing 113.6 kg will be prescribed a diet of 1500 to 1800 kcal/day. Meanwhile, all participants will be instructed to keep a daily food and calorie diary, and they will be instructed to engage in low-to-moderate intensity physical activities such as jogging and walking for at least 5 days per week and for at least 210 minutes per week, preferably 270 minutes per week.

All patients will be required to keep a diet and exercise diary at least 4 days per week. The intervention time for lifestyle intervention includes a 12-week treatment phase and a 12-week follow-up period.

#### 2.7.2. “Moxibustion for Harmonization of Yin and Yang” Group

Shenque (RN8) and Mingmen (DU4) will be chosen as acupoints (Figure 2). The acupoints are located in accordance with the national GB/T 12346–2006 acupoints standard [32]. Each treatment lasts 60 minutes once a week and alternates between “Wenyang Yishen moxibustion” and “Peiyuan Guben moxibustion.” For a total of 12 weeks, each patient received “WenYang Yishen moxibustion” followed by “Peiyuan Guben moxibustion.” The width and length of the patient's moxibustion site are measured using the same body measurement method before performing “Wenyang Yishen moxibustion.” We take about 700 g of fresh ground ginger with moderate dryness and wetness and shape it into a round cake with a diameter of about 20 cm and a thickness of about 2.5 cm on a sterile towel. We light 25 g of moxa with a diameter of about 18 cm on top of the ginger. When the bottom temperature reaches approximately 37°, the moxibustion materials can be applied to the patient's waist for treatment. The temperature should be kept between 43 and 45°, depending on the patient's tolerance. It is preferable to add the moxa after about 10 minutes of burning. When moxibustion occurs, there is a slight red burning heat in the patient's partial skin. Moxibustion takes 60 minutes. The operation of “Peiyuan Guben moxibustion” is the same as that of “WenYang Yishen moxibustion,” which is centered on Shenque. Moxa is selected from folium *artemisia argyi* from Qichun County, Hubei. We slice the fresh ginger and put it into a ginger grinder to crush it to make about 1 mm minced ginger. We take out the minced ginger and squeeze out the excess water to keep the ginger mud soft and moist. The humidity is controlled at 80–90% (measuring with a moisture tester). The prepared grated ginger is stored in a refrigerator at 4°C and heated in a microwave oven on medium-high heat for 5 minutes before applying moxibustion. During the moxibustion process, a digital thermometer will be placed between the sterile towel and the acupoint to control the moxibustion temperature.

#### 2.7.3. Gentle Moxibustion Group

In this group, Zhongwan (RN12), Guanyuan (RN4), and Sanyinjiao (SP6) will be selected (Figure 3). In order to keep the local skin's surface temperature at 45°C ± 2°C for 20 minutes, a lit moxa stick (1.5 cm diameter moxa cone grown in Qichun County, Hubei, China) will be placed 2–3 cm away from the skin. For 12 weeks straight, a gentle moxibustion procedure will be performed every other day, three times per week. During the menstrual cycle, the treatment will be postponed.

### 2.8. Outcome Measurements

During the screening period, all subjects will fill out a questionnaire about demographic data such as gender, age, nationality, education level, occupation, marital status, height, and weight, as well as disease situations such as time and duration. Before randomization, serum follicular production hormone (FSH) levels will be measured and analyzed. Before treatment (screening period, first visit), after treatment (4th week, 8th week, and 12th week), and at follow-up (18th week and 24th week), each participant will receive a clinical assessment of primary and secondary outcome measurements. If both of the participants' menopausal obesity meet the inclusion criteria, the menopausal obesity with the more severe symptoms will be evaluated.  Figure 4 depicts the timetable for this study.

#### 2.8.1. Primary Outcome Measurement

Since waist circumference is the easiest and most practical indicator to quantify obesity; evaluations will be done at weeks 0, 4, 8, 12, 18, and 24 to compare the rate of waistline reduction with the baseline. The correct method for waist circumference is to check the horizontal length of the huckle center or the lowest point of the ribs and the middle line of the outer horizontal line of the iliac crest. In order to avoid the errors generated during the measurement process, the test is measured by a professional training doctor.

#### 2.8.2. Secondary Outcome Measurement

1. Obesity-related indicators: weight (WG), body mass index (BMI), hip circumference (HC), waist-hip-ratio (WHR), and body fat percentage (F%) will be evaluated by Omron somatic fat scalea (HBF-219T) at weeks 0, 4, 8, 12, 18, and 24.
2. The Traditional Chinese Medicine clinical syndrome: the criteria for determining a diagnosis will be the TCM clinical syndrome scores. According to the 1997 5th National Obesity Research Conference's revisions to the diagnostic and treatment assessment criteria for simple obesity, lower scores indicate better physical conditions. The aggregate score runs from 0 to 30, and outcomes will be evaluated at weeks 0, 12, 18, and 24.
3. The Impact of Weight on Quality of Life Questionnaire (IWQOL-Lite): patients' levels of life quality improvement is measured using the IWQOL-Lite scale, and there is a significant negative correlation between this scale and single overall life satisfaction. The total score runs from 31 to 155, with lower numbers indicating a higher quality of life, and outcomes will be evaluated at weeks 0, 12, and 24.
4. The modified Kupperman score before and after treatment: the clinical symptoms of menopause are assessed using the modified Kupperman score. The total score runs from 0 to 63, with lower scores reflecting the lighter the patient's clinical symptoms; outcomes will be evaluated at weeks 0, 12, and 24.
5. The MOS Item Short from Health Survey (SF-36) scale: a widely accepted health-related quality of life assessment is the SF-36. Higher scores indicate greater living quality. The total score goes from 40 to 147; outcomes will be evaluated at weeks 0, 12, and 24.
6. Blood lipid-related indicators: low-density lipoprotein (LDL-C), high-density lipoprotein (HDL-C), cholesterol (TC), and triglyceride (TG) will be assessed at weeks 0 and 12, and the variation of the indicator is compared to baseline.
7. Estrogen-related indicators include estradiol (E2), and serum follicles to form hormone (FSH). If the patient still has menstruation when the blood test is taken, the test is performed on the 2nd or 3rd day and the corresponding treatment time is delayed. The change value of this indicator is compared to baseline; outcomes will be evaluated at weeks 0 and 12.
8. Health economics evaluation adopts cost-effective analysis, expressed in cost-effectiveness (COST/EFFECTIVESS, C/E).

### 2.9. Sample Size

Based on an examination of the available research, clinical knowledge, and consultation with clinical professionals, the mean improvement of the waist circumference was 6.15 ± 1.56 cm ($\bar{x}\pm S$) in the “moxibustion for harmonization of Yin and Yang” group and 3.94 ± 1.14 cm ($\bar{x}\pm S$) in the gentle moxibustion group. A total of 96 individuals are needed in each group to achieve a one-sided significance level of *α* = 0.025 and an 80% power. A total of 216 patients will be included in the study, with 108 individuals per treatment arm, assuming a 10% dropout rate.

### 2.10. Data Monitoring and Management

Print and digital case report forms will be used to maintain all data (CRFs). Primary entries cannot be modified, and any corrections require a signature in the appended comments along with an explanation. CRFs are only accessible to outcome assessors, and duplicate data input will be done. All facets of the company are under the control of the Wuhan research team. Every month, this experiment and its results will be monitored by the Hubei Provincial Hospital of TCM's ethics committee, which will also ultimately decide whether to end the trial. Interventionists will keep an eye out for negative situations and respond properly with advice and encouragement. The protocol requirements must be understood and followed by all researchers, acupuncturists, and related personnel.

### 2.11. Statistical Analysis

SAS 9.3 software will be used by an impartial statistician to analyze the data (SAS Institute Inc, Cary, NC). Any participant who completes the randomized stage and receives at least one intervention will be analyzed using a full analysis set (FAS), with missing data for the important outcomes interpolated with the last observation carried forward, in accordance with the intention-to-treat (ITT) analysis strategy. Multiple imputations will be used to deal with missing data. All statistical inspections were used for bilateral testing, and statistical significance will be determined at *P* < 0.05.

For the patient's missing data, it is assumed that the deletion data is randomly missing, the lacking value of the research main indicator is used for multiple filling methods, the stochastic missing deletion assumption of multiple filling is performed, and the stability test of the missing data filling results is carried out by using pattern mixture model (PMM). The measurement data is described by average ± standard deviation ($\bar{x}\pm S$), median, maximum, and minimum, and the counting data and grade data are described by cases and percentages. Intergroup comparison will select the analysis method according to the data distribution feature: the measurement data is used to test or nonparameter testing; the count data is used in*χ*^2^inspection or Fisher's exact probability method, and the grade data is used in the nonparameter test. Compared with the baseline value, the metering data is used in pair*T*inspection or nonparameter test, and counting materials use nonparameter test.

### 2.12. Safety Assessment

Vital signs and adverse events will be considered in the moxibustion safety evaluation. Prior to randomization and after therapy, a general physical examination using safety indicators such as blood pressure, heart rate, respiration, pulse, and body temperature will be performed. Aside from that, the frequency of adverse events, including moxibustion burns, blistering, dizziness, ulceration, infection, local abscess, irregular vaginal bleeding, fatigue, allergies, and anorexia will be meticulously recorded in the CRFs and monitored by the Ethics Committees.

### 2.13. Quality Control

The acupuncture, methodology, and statistics specialists examine and make revisions to the study protocol. A predetermined standard operating procedure will be used to teach the relevant employees. Through health education and prompt follow-up, patient compliance will be increased. If the subjects stop using moxibustion or depart from the procedure, the results will also be assessed by outcome assessors. This study will carry out a central randomization system to prevent bias in selection. At the same time, one of the most crucial strategies for preventing bias is the careful selection of inclusion and exclusion criteria, contributing to the objectivity of conclusions. A third-party blinded method will be applied to this study, namely, for assessing efficacy and safety by assessors who are not familiar with the group characteristics. To ensure the smooth progress of the study, all clinical researchers will be trained in the SOPs about moxibustion before the study begins to improve the consistency of researchers' and spectators' internal observations, in order to guarantee the validity of the conclusions. We will conduct sensitivity analyses in the per-protocol set. During this study, we will hold regular multicenter team meetings and go through routine checks to prevent center bias.

## 3. Discussion

The NCD risk factor collaboration [33] has shown that obesity is a significant worldwide health problem with a rise in prevalence from 3.1% in 2014 to 8.1% in 2018 [34]. It is estimated that 85 million Chinese adults aged 18–69 were obese in 2018 [35]. At present, the research on the treatment of obesity at domestic and abroad levels is mainly concentrated on acupuncture therapy, electroacupuncture, acupoint embedding, etc., with less research on moxibustion [36, 37]. Moxibustion, which comes in a variety of forms and is one of Traditional Chinese medicine's external therapeutic modalities, has been proved to be useful in the management of obesity [38–41], but it is considered to be a complementary therapy to acupuncture, which is usually used in combination with other therapeutic methods in clinical practice, resulting in the superiority of moxibustion being not fully realized. So far, few clinical trials have been conducted to confirm the efficacy and safety of moxibustion therapies for menopausal obesity. This is the first randomized controlled trial focusing on the variations in the effectiveness of “moxibustion for harmonization of Yin and Yang” compared to the gentle moxibustion for treating menopausal obesity. The outcomes will present evidence for better clinical effectiveness and prescription choice for moxibustion. Additionally, the outcomes of this experiment will be utilized to verify the safety and efficacy of the “moxibustion for harmonization of Yin and Yang” in regard to menopausal obesity treatment and provide high-level evidence-based evidence supporting the use of “moxibustion for harmonization of Yin and Yang” in the therapeutic treatment of menopausal obesity.

As stated by TCM's fundamental theory, the main causes of menopausal obesity are gradual failure of kidney qi, exhaustion of heavenly tenth, and Yin-Yang disharmony. The “moxibustion for harmonization of Yin and Yang” has the capacity to warm Yang and dredge collateral vessels, strengthen the root and reinforce deficiency, and mediate Yin and Yang; its thoughts originated from the theory of mutual rooting of Yin and Yang in classics of traditional Chinese medicine “Huangdi Neijing,” which is a detriment to yang affects yin and detriment to yin affects yang. When conducting syndrome differentiation and determining remedies, it pays close attention to the surroundings, individual constitution, and climatic and seasonal variables. By tonifying the pattern of dual deficiency of qi and blood, as well as Yin and Yang, eliminating the pathogenic factors of dampness and cold, the body functions will be in a state of Yin and Yang coordination and harmony. Hence, this study will select Shenque (RN8) and Mingmen (DU4) on the “moxibustion for harmonization of Yin and Yang” and Zhongwan (RN12), Guanyuan (RN4), and Sanyinjiao (SP6) on the gentle moxibustion because of the following reasons: (1) these acupoints have been demonstrated to be effective in accelerating metabolism and alleviating menopausal symptoms [25], (2) the gentle moxibustion candidate refers to the unified use of national Chinese medicine colleges, and the 13th five textbooks published by China Traditional Chinese Medicine “Acupuncture and Moxibustion Therapy” have pre- and postmenopausal symptoms and obesity-related prescriptions, and (3) one of the acupoints chosen is on the Yang side of the waist, the other is on the Yin side of the abdomen, and the two acupoints are located in the middle of the human body, reflecting the concept of “moxibustion for harmonization of Yin and Yang.”

From the following three perspectives, the efficacy evaluation will be carried out: obesity-related indicators, menopausal and obesity symptoms, and blood biological indicators. Waist circumference is a simple and important anthropometric measure of total and intra-abdominal body fat that the National Heart, Lung, and Blood Institute recommends as an indication of obesity in adults for the diagnosis, assessment, and treatment of overweight and obesity [42, 43]. Therefore, the primary outcome will be measured using the WC, which is valid, trustworthy, intuitive, and more accurate than the BMI in reflecting body adiposity [44]. At the same time, the obesity-related indicators (BMI, WG, HC, WHR, F%), obesity and menopause scale assessment (TCM clinical syndrome scores, modified Kupperman score, IWQOL-Lite, SF-36), and the changes in blood biochemical indicators (TC, TG, LDL-C, HDL-C, E2, FSH) will be assessed before and after therapy in this experiment as secondary outcomes. Patients with menopausal obesity have more serious symptoms and disturbed hormone levels [45]. Hence, IWQOL-LITE and SF-36 will be performed to assess symptoms and overall health of obesity [46, 47]. The Modified Kupperman score will be performed to identify patients with menopausal symptoms [48], and E2, and FSH will be used to assess the hormone levels in menopausal patients [49].

In conclusion, this multicenter, randomized, parallel, and controlled trial will evaluate the viability and superiority of “moxibustion for harmonization of Yin and Yang” and gentle moxibustion, as well as the efficacy and safety of various types of moxibustion treatments for menopausal obesity. It will also enhance the standardization of moxibustion for menopausal obesity and, to a greater extent, provide a clinical foundation for treatments, thereby better playing the role of moxibustion in disease treatment and health care.

## Figures and Tables

**Figure 1:** Flow chart.

**Figure 2:** Locations of acupoints in the “moxibustion for harmonization of Yin and Yang” group.

**Figure 3:** Locations of acupoints in the gentle moxibustion group.

**Figure 4:** Study schedule. IWQOL-Lite, the impact of weight on quality of life questionnaire; SF-36, the MOS item short from health survey; TCM, Traditional Chinese Medicine.

## Data Availability

Since no datasets were created or examined for this research, data sharing is not applicable.

## Abbreviations

WC: Waist circumference
WG: Weight
F%: Body fat percentage
BMI: Body mass index
HC: Hip circumference
WHR: Waist to hip ratio
ITT: Intention-to-treat
IWQOL-Lite: Impact of Weight on Quality of Life Questionnaire
SF-36: MOS item short from health survey
TC: Cholesterol
TG: Triglycerides
LDL-C: Low-density lipoprotein
HDL-C: High-density lipoprotein
E2: Estradiol
FSH: Serum follicle-forming hormone
STRICTA: Standards for reporting interventions for controlled trials of acupuncture
SPIRIT: Standard protocol items: recommendations for intervention trials
TCM: Traditional Chinese medicine.
